# Mathematical Modelling and Hierarchical Encourage Particle Swarm Optimization Genetic Algorithm for Jet Pipe Servo Valve

**DOI:** 10.1155/2022/9155248

**Published:** 2022-07-01

**Authors:** Jia Chen, Fei Li, Yi Yang, Yi Gao

**Affiliations:** ^1^School of Electronic Engineering, Xi'an Shiyou University, No. 18, East Section of Electronic 2nd Road, Xi'an, Shannxi, China; ^2^Shannxi Key Laboratory of Measurement and Control Theory for Oil and Gas Wells, Xi'an, Shannxi, China

## Abstract

The jet pipe servo (JPS) valve is one key component, whose dynamic performance directly influences the aircraft's maneuverability. In this paper, a more accurate mathematical model and a novel multiobjective hierarchical encourage particle swarm optimization genetic algorithm (HEPGA) are proposed to improve the dynamic performance of the jet pipe servo valve. By optimizing the main structure parameters of the jet pipe servo valve, the adjustment and overshoot in the dynamic performance are reduced by 24.28% and 51.39%, respectively, compared with the prototype before optimization. To obtain a more accurate mathematical model, the computational fluid dynamics (CFD) is introduced to modify the analytical model considering the turbulent submerged free jet. Different from conventional numerical simulation, the dynamic mesh technique is used to analyze the flow field distribution by considering the force interaction of various parts of the jet pipe servo valve under actual working condition. Then, the HEPGA with better convergence is utilized because of the conflict of adjustment and overshoot. This proposed hybrid algorithm introduces the concept of staff welfare system to divide the population into elite individuals and excellent individuals of particle swarm optimization and general individuals of genetic algorithm. Meanwhile, the convergency performance of the HEPGA is evaluated through the Rosenbrock function by comparing with other particle swarm genetic hybrid methods. Subsequently, the experimental platform is constructed and the dynamic performance tests are conducted on the prototype after optimization. The experimental results verify the accuracy of the established mathematical model and the significant improvement of dynamic performance of the jet pipe servo valve.

## 1. Introduction

The JPS valve, which is a core component of electro-hydraulic servo system, is widely concerned and applied in the aerospace system because of its antipollution, high sensitivity, and long service life [1–3]. Especially, the JPS valve has better antipollution performance and higher reliability than the nozzle flapper valve [4–6].

Due to the excellent performance, many scholars around the world have studied and improved the jet pipe servo valve. Henri et al. [1] established a nonlinear dynamic model of the jet pipe, and revealed that the nonlinear mechanical of jet pipe is the major factor of hysteresis. Finite element analysis (FEA) was utilized to calculate feedback force of the feedback rod when the torque motor is input control current [2]. An analytical model of the torque motor was deduced by using the equivalent magnetic circuit model, and verified by the numerical simulation [4]. When current is input to the torque motor, the armature assembly rotates under the action of the electromagnetic force. Then the dynamic performance of the armature assembly was investigated by establishing the mathematical model which is verified by FEA [5]. The comparison results show that the error between the established model and numerical simulation is 6.6%. The rotation of the armature drives the jet pipe to deflect to provide different hydrodynamic energy to the two receivers. The jet pipe and the two receivers constitute the jet pipe amplifier which is the crucial part of the JPS valve.

With the development of computer, computational fluid dynamics (CFD) acquires widespread application in the fluid field analysis of different valves [6–10]. Especially for the complex flow field in the jet tube amplifier, it needs to be analyzed with the CFD. Li [11] utilized the CFD results of the static pressure analysis of the prestage to modify the mathematical model based on the turbulent submerged jet theory. Because the jet pipe has been rotating as the valve works, the transient flow field was analyzed in the prestage by using dynamic mesh technique [12]. Meanwhile, the laminar and turbulent flow state in the JPS valve were considered together to build a mathematical of the jet pipe amplifier [13]. The pressure oscillations in the jet pipe amplifier were investigated by using CFD [14, 15], which present that the main source of the pressure oscillations is derived from cavitation and shear layer instability. These studies have contributed to improve the performance of jet pipe amplifier. Unfortunately, the flow field distribution of the jet pipe amplifier has not been studied when the JPS valve is in the operating mode, where the flow field distribution is more complicated.

To improve the dynamic performance of the JPS valve, the scholars above have devoted themselves to research the valve's components including torque motor, armature assembly, and jet pipe amplifier. Unfortunately, very few documents on the dynamic performance of the JPS valve have been published publicly. In paper [16, 17], a multidomain model of the JPS valve was proposed, and the relationship of the load flow rate and the nozzle displacement is written as a proportional relationship. By using the Bernoulli's equations, a dynamic model of the JPS valve was built to analyze reliability [3]. The established mathematical model of the whole JPS valve neglects the submerged jet characteristic.

Thus, a more accurate mathematical model of the JPS valve is needed to be developed to analyze the valve's dynamic characteristics which are the main purpose of the above researches. The dynamic characteristics are composed of steady-state error, overshoot, and adjustment time in step response. And the overshoot and the adjustment time are always to be expected as small as possible in system design. However, the two performance indicators are in in conflict. In other words, the reduction of the overshoot will increase the adjustment time. Alternatively, the reduction of the adjustment will increase the overshoot.

To satisfy the two objectives simultaneously, a multiobjective optimization algorithm is needed to optimize the main structure parameters of the jet pipe servo valve. Genetic algorithm (GA) and particle swarm optimization (PSO) have acquired successful application in the multiobjective optimization [18, 19]. To improve the efficiency and convergence, scholars always combine the two algorithms [20–30]. There are mainly four methods to implement such connections. The first hybrid method utilizes the genetic operation to update the particle's velocity and position, which is called substituted method [20]. In this method, the PSO is the main body of the optimization algorithm, where the GA cannot be used to the best advantage. In other words, the two optimization algorithms enjoy different status. Then, the parallel method and the sequential method acquire their applications, where the GA and the PSO have same status. In the parallel method, the population is divided into two parts, one for GA operation and the other for PSO operation. The individuals operated by the evolutionary algorithm are recombined to form an update population in the next iteration and divided again to implement the GA and the PSO operations, respectively [21–24]. And for the sequential method, all the individuals utilize the GA and the PSO algorithm to generate the new population of next iteration [25–28]. These two methods still have deficiencies. The PSO individuals of the parallel method is easy to fall into local optimum, while in the sequential method, the GA operation is required for all individuals, which takes a long calculation time. Ultimately, the fourth method introduces other algorithms, such as fuzzy approach, or uses more complex hybrid structure. For instance, in the method of introducing other algorithms, a fuzzy system is applied to change the influence factor in the GA and PSO, where the hybrid structure still utilizes the sequential method [29]. In the paper [30], the parallel method is firstly utilized to classify the population to implement the crossover and the PSO operations, respectively, and then all the individuals are performed the same mutation rate. The results of this complex hybrid method show better performance. However, the elite individuals from the PSO operation are easy to lose competitive advantage by the same mutation operation. Therefore, this paper proposes a novel hierarchical encourage particle swarm genetic algorithm, which divides the population more exactly and utilizes different mutation rates to protect the excellent individuals and ensure the diversity.

To sum up, this paper is organized as follows. The working principle of the JPS valve is described in Section 2.  Section 3 derives the mathematical model of the JPS valve by considering the turbulent submerged jet. To modify the dynamic model, Section 4 analyzes the stiffness of the complex feedback rod and the flow filed of the jet pipe amplifier in actual working condition.  Section 5 introduces the structure of the novel hierarchical encourage particle swarm genetic algorithm and verify its advantage.  Section 6 presents the experimental platform which is used to verify the mathematical model and the effectiveness of the proposed optimal algorithm. Finally, the dynamic performance of the optimal jet pipe servo valve is compared to the experimental results and the dynamic performance before optimization in Section 7.

## 2. Working Principle of the Jet Pipe Servo Valve

As shown in Figure 1, the JPS valve includes torque motor, armature assembly, jet pipe amplifier, and spool valve. The magnet part of the torque motor forms a closed-loop magnetic circuit, which generates inherent magnetic flux with equal size and same direction in the four air gaps. As the current is input into the control coil, the control magnetic flux with equal size and opposite direction is generated. Then the electromagnetic force drives the armature assembly to rotate around the armature's center. Accordingly, the jet tube fixed on the armature deflects.

The deflection of the jet tube causes the overlapping area of the jet nozzle and one receiving hole to be greater than that of the jet nozzle and the other receiving hole. Therefore, the flow rate injected into one receiving is greater than that of the other receiving hole when high-pressure oil is ejected from the jet nozzle. Since the two receiving holes connect with the control chambers at both ends of the spool valve, respectively, the high-pressure oil entering the two receiving holes forms a differential pressure at both ends of the spool. And the differential pressure drives the spool to move in the opposite direction of the deflection of the jet tube. The movement of the spool valve leads to the change of the direction of the high-pressure oil. Meanwhile, the feedback rod connecting with the center of the spool valve and the spring tube generate feedback torque, respectively. When the control torque of the torque motor is equal to the feedback torque the spool valve is stable. Afterwards the servo valve outputs the proportional flow rate or pressure according to the control current.

## 3. Dynamic Model of the JPS Valve

### 3.1. Torque Motor

The electromagnetic force applied on the armature is controlled by changing the values of the control magnetic flux in the torque motor, which can be expressed as

(1) $$\begin{array}{c} F=5.1\times 10^{-8}U^{2}\frac{\text{d}G}{\text{d}x}. \end{array}$$

Equation (1) is Maxwell's electromagnetic force formula, where *F* is the electromagnetic force, *U* is the magnetic pressure drop, *G* is the magnetic conductivity, and *x*_*g*_ is the displacement of the armature.

As shown in Figure 2, when the control coil is given the negative current, the direction of the control magnetic flux and the inherent magnetic flux in the air gap *a* and *d* is the same, while that in the air gap *b* and *c* is the opposite. Thus, the electromagnetic suction force in the air gap *a* and *d* is greater than that in the air gap *b* and *c*. According to equation (1), the electromagnetic suction forces in air gaps can be written as

(2) $$\begin{array}{c} F_{1}=5.1\times 10^{-8}{\left(\frac{B_{p}h_{g}}{\mu_{0}}+\frac{B_{c}h_{g}}{\mu_{0}}\right)}^{2}\frac{\mu_{0}A_{g}}{{\left(h_{g}-x_{a}\right)}^{2}}. \end{array}$$

(3) $$\begin{array}{c} F_{2}=5.1\times 10^{-8}{\left(\frac{B_{p}h_{g}}{\mu_{0}}-\frac{B_{c}h_{g}}{\mu_{0}}\right)}^{2}\frac{\mu_{0}A_{g}}{{\left(h_{g}+x_{a}\right)}^{2}}. \end{array}$$

As shown in Equations (2) and (3), *F*_1_ and *F*_2_ are the electromagnetic suction forces in the air gap *a* and *b*, respectively. *h*_*g*_ is the thickness of the air gap when the armature has no rotation. *A*_*g*_ is the area of magnetic pole surface. Since the armature's rotation angle is so small that the rotation angle can be expressed as *x*. *B*_*p*_ is the inherent magnetic density, and *B*_*c*_ is the control magnetic density. *μ*_0_ is the air magnetic conductivity coefficient.

The electromagnetic suction forces drive the armature to rotate, resulting in the generation of electromagnetic torque. Due to the distance *a* from the armature's center to the center of the air gap, the electromagnetic torque can be written as

(4) $$\begin{array}{c} T_{d}=2aF_{1}-2aF_{2}. \end{array}$$

Introducing Equations (2) and (3) into Equation (4), respectively, the electromagnetic torque can be expressed as

(5) $$\begin{array}{c} T_{d}=\frac{10.2a\times 10^{-8}}{{\left[1-{\left(x_{a}/h_{h}\right)}^{2}\right]}^{2}}\left\{\frac{4B_{p}^{2}A_{g}x_{a}}{\mu_{0}g}\left[1+{\left(\frac{B_{c}}{B_{p}}\right)}^{2}\right]+\frac{4B_{p}B_{c}A_{g}}{\mu_{0}}\left[1+{\left(\frac{x_{a}}{h_{g}}\right)}^{2}\right]\right\}, \end{array}$$

where to improve the linear characteristics of the torque motor, the armature's displacement *x*_*a*_ is designed to be less than three times the air gap *g*. Then the item (*x*_*a*_/*h*_*g*_)^2^ can be considered to be much less than 1. Similarly, to prevent the control flux from weakening the magnetism of the permanent magnet, the inherent magnetic density *B*_*p*_ needs to be much smaller than the control magnetic density *B*_*c*_. Therefore, Equation (5) can be written as

(6) $$\begin{array}{c} T_{d}=\frac{40.8a\times 10^{-8}B_{p}^{2}A_{g}x_{a}}{\mu_{0}g}+\frac{40.8\times 10^{-8}B_{p}B_{c}A_{g}}{\mu_{0}}. \end{array}$$

Meanwhile, the control magnetic density *B*_*c*_ is proportional to the number of coil turns *N*_*c*_ and control current *i*_*c*_. Then the electromagnetic torque can be expressed as

(7) $$\begin{array}{c} T_{d}=K_{a}x_{a}+K_{t}i_{c}, \end{array}$$

where *K*_*a*_=40.8*a* × 10^−8^*B*_*p*_^2^*A*_*g*_/*μ*_0_*h*_*g*_ and *K*_*t*_=20.4 × 10^−8^*B*_*p*_*A*_*g*_*aN*_*c*_/*h*_*g*_.

### 3.2. Armature Assembly

The torque motor drives the armature assembly to rotate by an angle *θ*, the value of which is such small as can be written as

(8) $$\begin{array}{c} \theta_{a}=\frac{x_{a}}{a}. \end{array}$$

The spring tube with upper end fixed on the armature is nested in the ring at the top of the feedback rod, as shown in Figure 3(a). Due to the rotation of the armature and the displacement of the feedback rod *x*_*v*_, the mass center of the spring tube has translational displacement *x*_*g*_. Then the top of the spring tube has displacement *x*_*t*_.

(9) $$\begin{array}{c} x_{t}=x_{g}+r_{1}\theta_{a}, \end{array}$$

where *r*_1_ is the distance from the mass center of the spring tube to the armature's center.

The spring tube fixed at the upper end is considered as a cantilever beam, the spring coefficient of which can be acquired by the following equation:

(10) $$\begin{array}{c} \left\{\begin{array}{c} K_{11}=\frac{EI}{\left(L^{3}/12\right)},\\ K_{12}=K_{21}=\frac{EI}{\left(-L^{2}/6\right)},\\ K_{22}=\frac{EI}{\left(L/4\right)}, \end{array}\right. \end{array}$$

where *E* is the Young's modulus of the spring tube, *I* is the moment of inertia of the spring tube, *L* is the length of the spring tube, and *K*_11_, *K*_12_, *K*_21_, and *K*_22_ are the spring coefficients of the spring tube.

Then the force *F*_tube_ and the torque *T*_tube_, respectively, generated by the spring tube can be written as

(11) $$\begin{array}{c} \left\{\begin{array}{c} F_{\text{tube}}=K_{11}x_{t}+K_{12}\theta_{a},\\ T_{\text{tube}}=K_{21}x_{t}+K_{22}\theta_{a}. \end{array}\right. \end{array}$$

As illustrated in Figure 3(a), the deflection of the spring tube applies force on the feedback rod. When the spool moves, the bottom end of the feedback rod is affected by the force of the spool at the same time. Thus, the displacement of the rod's bottom end is

(12) $$\begin{array}{c} x_{g}-\left(r+b\right)\theta_{a}-x_{v}. \end{array}$$

Due to the deformation of the feedback rod, the feedback force and the feedback torque can be expressed as

(13) $$\begin{array}{c} \left\{\begin{array}{c} F_{f}=K_{f}\left[\left(r+b\right)\theta_{a}+x_{v}-x_{g}\right],\\ T_{f}=K_{f}\left[\left(r+b\right)\theta_{a}+x_{v}-x_{g}\right]\left(r+b\right), \end{array}\right. \end{array}$$

where *F*_*f*_ is the feedback force, *T*_*f*_ is the feedback torque, and *K*_*f*_ is the spring coefficient of the feedback rod.

There is interaction force between armature, spring tube, and feedback rod, which can form armature-rod assembly. Based on the interaction of force and torque, the equilibrium equations of force and torque applied on the armature-rod assembly can be obtained by

(14) $$\begin{array}{c} \left\{\begin{array}{c} F_{f}=m_{a}{\overset{¨}{x}}_{g}+B_{a}{\dot{x}}_{g}+F_{\text{tube}}+F_{\text{flow}},\\ T_{d}=J_{r}{\overset{¨}{\theta }}_{a}+B_{r}{\dot{\theta }}_{a}+T_{\text{tube}}+T_{f}-T_{\text{flow}}, \end{array}\right. \end{array}$$

where *m*_*a*_ is the mass of the armature-rod assembly, *B*_*a*_ is the damping coefficient for the translation of the armature-rod assembly, *J*_*r*_ is the moment inertia of the armature-rod assembly, *B*_*r*_ is the damping coefficient for the rotation of the armature-rod assembly, *F*_flow_ is the force generated by the reflected flow from two receiver holes, and *T*_flow_ is the torque generated by the force *F*_*flow*_.

From Equations (7) to (14), the differential equation of input current, armature rotation angle, and spool displacement can be expressed as

(15) $$\begin{array}{c} K_{t}\left(m_{a}{\overset{¨}{i}}_{c}+B_{a}{\dot{i}}_{c}+K_{f}i_{c}+K_{11}i_{c}\right)=J_{r}m_{a}{\ddddot{\theta }}_{a}+\left(J_{r}B_{a}+B_{r}m_{a}\right){\dddot{\theta }}_{a}+\left(J_{r}K_{f}+J_{r}K_{11}+B_{r}B_{a}\right){\overset{¨}{\theta }}_{a}+B_{r}\left(K_{f}+K_{11}\right){\dot{\theta }}_{a}\\ +B_{a}\left[K_{21}r+K_{22}+K_{f}{\left(r+b\right)}^{2}-K_{\theta }\right]{\dot{\theta }}_{a}+\left[K_{21}r+K_{22}+K_{f}{\left(r+b\right)}^{2}-K_{\theta }\right]\left(K_{f}+K_{11}\right)\theta_{a}+K_{f}\left(r+b\right)m_{a}{\overset{¨}{x}}_{v}\\ +K_{f}B_{a}\left(r+b\right){\dot{x}}_{v}+K_{f}\left(r+b\right)\left(K_{f}+K_{11}\right)x_{v}-\left[K_{21}-K_{f}\left(r+b\right)\right]F_{\text{flow}}-m_{a}{\overset{¨}{T}}_{\text{flow}}-B_{a}{\dot{T}}_{\text{flow}}-\left(K_{f}+K_{11}\right)T_{\text{flow}}. \end{array}$$

### 3.3. Jet Pipe Amplifier

When the flow is ejected from the jet pipe amplifier, the high-pressure energy of the fluid is converted into the kinetic energy of the fluid. Due to the deflection of the nozzle, the flow rate of high-speed fluid entering the two receiving holes is different. As shown in Figure 4, the flow rate of flow into the right receiving hole is greater than that into the left receiving hole. Thus the pressure in the right receiving hole will be larger than that in the left receiving hole. Then the differential pressure will drive the spool to move towards the left direction, which is the opposite direction of the nozzle's deflection.

#### 3.3.1. Turbulent Submerged Jet Free Stream

The fluid is ejected from the nozzle into the fluid of the same density, which is named as submerged free jet stream [6]. As shown in Figure 5, due to the boundary entrainment, the free jet experiences a length *L*_0_ of decreasing in constant velocity region, and the constant velocity region is called as potential core. The diameter of the nozzle, the velocity distribution in the nozzle, and the Reynolds number all affect the potential core length *L*_0_, and the diameter of the nozzle *D*_*j*_ is the dominant influence [11]. The influence of the velocity distribution in the nozzle and the Reynolds number is neglected, and the potential core length *L*_0_ is supposed as [11]

(16) $$\begin{array}{c} L_{0}\approx 4.19D_{j}. \end{array}$$

To improve the efficiency of jet energy utilization, the vertical distance from nozzle exit to receiver *l*_*j*_ should be less than the potential core length *L*_0_. As shown in Figure 5, the diameter of the potential core *D*_*pf*_ with the geometric relationship with the distance *l*_*j*_ and the length *L*_0_ can be expressed as

(17) $$\begin{array}{c} D_{pf}\approx \frac{L_{0}-l_{j}}{4.19}=\frac{4.19D_{j}-l_{j}}{4.19}=D_{j}-\frac{l_{j}}{4.19}. \end{array}$$

To express concisely the diameter of the potential core *D*_*pf*_, the relative distance *λ*_*j*_=*l*_*j*_/*D*_*j*_ is introduced into Equation (16), and the diameter of the potential core *D*_*pf*_ is written as

(18) $$\begin{array}{c} D_{pf}=D_{j}\left(1-0.2387\lambda_{j}\right). \end{array}$$

Also, the diameter of turbulent mixing zone is given by

(19) $$\begin{array}{c} D_{tm}=D_{j}\left(1+2\lambda_{j}\tan\theta_{j}\right). \end{array}$$

When a bunch of flow with diameter *D*_*pf*_ shoots into an enclosed receiver hole, and the momentum of this bunch of flow equals a bunch of flow with velocity *u*_*j*_ and equivalent diameter *D*_*ij*_. As shown in Equation (17), the equivalent diameter is given by

(20) $$\begin{array}{c} D_{ij}=D_{j}\left(1-\psi \lambda_{j}\right), \end{array}$$

where *ψ* is the coefficient of flow pattern, which is supposed as [11]

(21) $$\begin{array}{c} \psi =\frac{1+0.4251\lambda_{j}-\sqrt{D_{r}/D_{j}}}{2.78\lambda_{j}}, \end{array}$$

where *D*_*r*_ is the diameter of one receiver hole.

Figure 4 shows that the two receiver holes and the nozzle have overlapping areas that receive the kinetic flow from the nozzle, respectively. Because the receiver hole with circular cross-sectional area of the channel has an included angle *θ*_*r*_ with the vertical direction, the shape of the receiver hole projected on the receiver's surface is elliptical. If the projection of the two receiver holes on receiver surface is assumed as circular, the area of the circular should be equal to the area of the elliptical. Then the relation of the two areas can be written as

(22) $$\begin{array}{c} \pi R_{el}^{2}=\pi \frac{R_{r}^{2}}{\cos\theta_{r}}, \end{array}$$

where *R*_*el*_ is the radius of the equivalent and *R*_*r*_ is the radius of the receiver hole.

Before the optimization, *θ*_*r*_ is set as 15°. The assumption error calculation is given by

(23) $$\begin{array}{c} R_{el}=\frac{R_{r}}{\sqrt{\cos15^{{}^{\circ}}}}=1.0175R_{r}. \end{array}$$

From Equation (23), when *R*_*r*_ is utilized to calculate the flow area of the receiver hole, the calculation error is less than 1.75% if *θ*_*r*_ is less than 15°.

#### 3.3.2. Calculation of the Flow Area

When the nozzle deflects towards the *x*-axis direction, the two shaded zones shown in Figure 4 are the receiving zones where the two receiver holes obtain the jet flow bunch, respectively. As shown in Figure 4, the area of the right receiver hole receiving jet flow from the nozzle is *A*_1_, which is given by

(24) $$\begin{array}{c} A_{1}\left(x_{j}\right)=S_{sector-o_{r1}MN}+S_{sector-o_{j}MN}-S_{o_{r1}Mo_{j}N}, \end{array}$$

where *S*_*sector*−*o*_*r*1_*MN*_ is the area of sector *O*_*r*1_*MN*, *S*_*sector*−*o*_*j*_*MN*_ is the area of sector *O*_*j*_*MN*, *S*_*o*_*r*1_*Mo*_*j*_*N*_ is the area of quadrangle *O*_*r*1_*MO*_*j*_*N*, and *x*_*j*_ is the displacement of the nozzle. According to the geometric relationship in Figure 3(b), *x*_*j*_ is given by

(25) $$\begin{array}{c} x_{j}=r\theta_{a}. \end{array}$$

Based on the geometrical relationship shown in Figure 4, the area of the shaded part on the right receiver hole can be written as

(26) $$\begin{array}{c} A_{1}\left(x_{j}\right)=R_{r}^{2}\theta_{1}+R_{j}^{2}\theta_{2}-\sin\theta_{1}R_{r}\left(R_{r}+0.5d-x_{j}\right), \end{array}$$

where *R*_*j*_ is the radius of the nozzle, *d* is the distance between the two receiver holes, *θ*_1_ is defined as ∠*Mo*_*r*1_*o*_*j*_, *θ*_2_ is defined as ∠*No*_*j*_*o*_*r*1_. According to the triangle cosine theorem, the angle *θ*_1_ and the angle *θ*_2_ can be obtained as

(27) $$\begin{array}{c} \theta_{1}=\arccos\frac{R_{r}^{2}+{\left(R_{r}+0.5d-x_{j}\right)}^{2}-R_{j}^{2}}{2R_{r}\left(R_{r}+0.5d-x_{j}\right)},\\ \theta_{2}=\arccos\frac{r_{j}^{2}+{\left(R_{r}+0.5d-x_{j}\right)}^{2}-R_{r}^{2}}{2r_{j}\left(R_{r}+0.5d-x_{j}\right)}. \end{array}$$

The area of the right receiver hole is composed of *A*_1_ and *A*_3_; hence,

(28) $$\begin{array}{c} A_{3}\left(x_{j}\right)=\pi R_{r}^{2}-R_{r}^{2}\theta_{1}-R_{j}^{2}\theta_{2}+\sin\theta_{1}\;R_{r}\left(R_{r}+0.5d-x_{j}\right). \end{array}$$

Similarly, *A*_2_ and *A*_4_ are given by

(29) $$\begin{array}{c} A_{2}\left(x_{j}\right)=R_{r}^{2}\theta_{3}+R_{j}^{2}\theta_{4}-\sin\theta_{3}\;R_{r}\left(R_{r}+0.5d+x_{j}\right),\\ A_{4}\left(x_{j}\right)=\pi R_{r}^{2}-R_{r}^{2}\theta_{3}-R_{j}^{2}\theta_{4}+\sin\theta_{3}\;R_{r}\left(R_{r}+0.5d+x_{j}\right), \end{array}$$

where *θ*_3_ is defined as ∠*M*′*o*_*r*2_*o*_*j*_ and *θ*_4_ is defined as ∠*N*′*o*_*j*_*o*_*r*2_. Applying the triangle cosine theorem, the angle *θ*_3_ and the angle *θ*_4_ are given by

(30) $$\begin{array}{c} \theta_{3}=\arccos\frac{R_{r}^{2}+{\left(R_{r}+0.5d+x_{j}\right)}^{2}-R_{j}^{2}}{2R_{r}\left(R_{r}+0.5d+x_{j}\right)},\\ \theta_{4}=\arccos\frac{R_{j}^{2}+{\left(R_{r}+0.5d+x_{j}\right)}^{2}-R_{r}^{2}}{2R_{j}\left(R_{r}+0.5d+x_{j}\right)}. \end{array}$$

To simplify calculation, the models of *A*_1_, *A*_2_, *A*_3_, and *A*_4_ are linearized as follows:

(31) $$\begin{array}{c} A_{1}\left(x_{j}\right)=A_{1}\left(0\right)+\alpha_{a1}x_{j},\\ A_{2}\left(x_{j}\right)=A_{2}\left(0\right)-\alpha_{a1}x_{j},\\ A_{3}\left(x_{j}\right)=A_{3}\left(0\right)-\alpha_{a2}x_{j},\\ A_{4}\left(x_{j}\right)=A_{4}\left(0\right)+\alpha_{a2}x_{j}. \end{array}$$

where *A*_1_(0), *A*_2_(0), *A*_3_(0), and *A*_4_(0) are the flow areas when the nozzle is in the middle between the two receiving holes, *α*_*a*1_ and *α*_*a*2_ are the area gradient. To compare the errors between the linear model and the nonlinear model, the relation curve between the area of the shaded part and the displacement of the nozzle is shown in Figure 6.

As shown in Figure 6, around the zero point of the nozzle displacement, the flow area of the linear model is close to the nonlinear model. Meanwhile, the JSP usually works near the zero point. Therefore, the linear model of the flow area can be used in the working condition.

Because of the symmetry of the cross-sectional area of the nozzle and the receiving hole, *A*_1_(0), *A*_2_(0), *A*_3_(0), and *A*_4_(0) have the following relationship:

(32) $$\begin{array}{c} A_{1}\left(0\right)=A_{2}\left(0\right),\\ A_{3}\left(0\right)=A_{4}\left(0\right). \end{array}$$

Then, the area gradient can be written as

(33) $$\begin{array}{c} \alpha_{a1}=\frac{A_{2}\left(0\right)}{r_{j}-0.5d}=\frac{R_{er}^{2}\theta_{3}+r_{j}^{2}\theta_{4}-\sin\theta_{3}R_{er}\left(R_{er}+0.5d\right)}{r_{j}-0.5d},\\ \alpha_{a2}=\frac{A_{4}\left(0\right)-\pi R_{er}^{2}}{r_{j}-0.5d}=\frac{-R_{er}^{2}\theta_{3}-r_{j}^{2}\theta_{4}+\sin\theta_{3}\;R_{er}\left(R_{er}+0.5d\right)}{r_{j}-0.5d}. \end{array}$$

Due to the distance *l*_*j*_ between the nozzle and the surface of the receivers, the calculation of the overlapping areas *A*_1_ and *A*_2_ should consider the submerged free jet stream theory. From Equation (20), the overlapping areas can be expressed as

(34) $$\begin{array}{c} A_{i1}\left(x_{j}\right)=A_{1}{\left(1-\psi \lambda_{j}\right)}^{2}. \end{array}$$

(35) $$\begin{array}{c} A_{i2}\left(x_{j}\right)=A_{2}{\left(1-\psi \lambda_{j}\right)}^{2}. \end{array}$$

Then, Equations (24) and (26) are revised as

(36) $$\begin{array}{c} A_{3}\left(x_{j}\right)=\pi R_{r}^{2}-A_{1}{\left(1-\psi \lambda_{j}\right)}^{2},\\ A_{4}\left(x_{j}\right)=\pi R_{r}^{2}-A_{2}{\left(1-\psi \lambda_{j}\right)}^{2}. \end{array}$$

#### 3.3.3. Energy Conversion in the Receiver

The volume flow rate *q*_*j*_ through the nozzle can be written as

(37) $$\begin{array}{c} q_{j}=C_{dj}A_{j}\sqrt{\frac{2\left(P_{s}-P_{0}\right)}{\rho }}, \end{array}$$

where *C*_*dj*_ is the coefficient of nozzle, *ρ* is the fluid's density, *A*_*j*_ is the cross-sectional area of the nozzle, *P*_*s*_ is the high-pressure from the top of the jet tube, and *P*_0_ is the outlet pressure of the nozzle.

Because the outlet pressure *P*_0_ is much lower than the high-pressure from the top of the jet tube, *P*_0_ can be neglected. Hence, the velocity of free jet at the nozzle exit is given by

(38) $$\begin{array}{c} u_{j}=\frac{q_{j}}{A_{j}}=C_{dj}\sqrt{\frac{2\left(P_{s}-P_{0}\right)}{\rho }}\approx C_{dj}\sqrt{\frac{2P_{s}}{\rho }}. \end{array}$$

If the fluid is assumed to be incompressible, the force applied on the fluid in the receiver hole can be calculated by the momentum equation of free jet impinging on the equivalent moving mechanical piston (EMMP), as shown in Figure 7. In time interval d*t*, the mass *m*_*j*_ of flow impinging on the EMMP can be written as

(39) $$\begin{array}{c} dm_{j}=\rho A_{i1}\left(u_{j}-u_{r}\cos\theta_{r}\right)\text{d}t, \end{array}$$

where *u*_*r*_ is the velocity of the EMMP.

When the free jet flow impinges on the EMMP, a part of flow is reflected at velocity *u*_01_, and the mass of this part of flow is given by

(40) $$\begin{array}{c} dm_{01}=\rho \left(A_{r}-A_{i1}\right)\left(u_{01}+u_{r}\right)\text{d}t. \end{array}$$

The fluid with mass (*dm*_*j*_ − *dm*_01_) moves with the EMMP at the velocity *u*_*r*_ after colliding with the piston. Based on the momentum theorem, the force of the jet flow acting on the EMMP can be expressed as

(41) $$\begin{array}{c} F_{j1}=\frac{dm\overset{⟶}{V}}{dt}=\left[\left(dm_{j}-dm_{01}\right)u_{r}\cos\theta_{r}-u_{01}dm_{01}+mu_{r}\right]-\left(u_{j}\cos\theta_{r}dm_{j}+mu_{r}\right)\\ =\left(dm_{j}-dm_{01}\right)u_{r}-u_{01}dm_{01}-u_{j}\cos\theta_{r}dm_{j}. \end{array}$$

Substituting Equations (39) and (40) into Equation (41), the force applied on the EMMP can be written as

(42) $$\begin{array}{c} F_{j1}=\rho A_{i1}{\left(u_{j}\cos\theta_{r}-u_{r}\right)}^{2}+\rho \left(A_{r}-A_{i1}\right){\left(u_{01}+u_{r}\right)}^{2}. \end{array}$$

Thus, the pressure caused by the force *F*_*j*1_ is given by

(43) $$\begin{array}{c} P_{r1}=\frac{F_{j1}}{A_{r}}=\frac{\rho }{A_{r}}\left[A_{i1}{\left(u_{j}\cos\theta_{r}-u_{r}\right)}^{2}+\left(A_{r}-A_{i1}\right){\left(u_{01}+u_{r}\right)}^{2}\right]. \end{array}$$

The volume flow rate into the spool valve can be written as

(44) $$\begin{array}{c} q_{L}=C_{dr}A_{r}\sqrt{\frac{2}{\rho }\left(P_{r1}-P_{1}\right)}. \end{array}$$

where *C*_*dr*_ is the flow coefficient of the receiver hole.

Then the pressure acting on the right end of the spool is given by

(45) $$\begin{array}{c} P_{1}=P_{r1}-\frac{q_{L}^{2}\rho }{2C_{dr}A_{r}^{2}}. \end{array}$$

Based on the principle of flow continuity in the right receiving hole, the velocity of the reflected flow *u*_01_ can be written as

(46) $$\begin{array}{c} u_{01}=\frac{u_{j}\cos\theta_{r}A_{i1}-u_{r}A_{r}}{A_{r}-A_{i1}}. \end{array}$$

Substituting Equation (43) into Equation (45), *P*_1_ is given by

(47) $$\begin{array}{c} P_{1}=\rho \left[\frac{A_{i1}{\left(u_{j}\cos\theta_{r}-u_{r}\right)}^{2}}{A_{r}-A_{i1}}-\frac{q_{L}^{2}}{2C_{dr}A_{r}}\right]. \end{array}$$

Due to the left movement of the spool, the EMMP in the left receiver hole moves at the same velocity *u*_*r*_. Hence, the mass of free jet flow impinging on the EMMP in time interval d*t* is given by

(48) $$\begin{array}{c} dm_{j2}=\rho A_{i2}\left(u_{j}\cos\theta_{r}+u_{r}\right)\text{d}t. \end{array}$$

The mass of flow reflected in time interval d*t* is given by

(49) $$\begin{array}{c} dm_{02}=\rho \left(A_{r}-A_{i2}\right)\left(u_{02}-u_{r}\right)dt. \end{array}$$

The force of free jet flow acting on the EMMP can be written as

(50) $$\begin{array}{c} F_{j2}=\rho A_{i2}{\left(u_{j}\cos\theta_{r}+u_{r}\right)}^{2}+\rho \left(A_{r}-A_{i2}\right){\left(u_{02}-u_{r}\right)}^{2}. \end{array}$$

The pressure generated by the force of the jet flow impinging is given by

(51) $$\begin{array}{c} P_{r2}=\frac{F_{j2}}{A_{r}}=\frac{\rho }{A_{r}}\left[A_{i2}{\left(u_{j}\cos\theta_{r}+u_{r}\right)}^{2}+\left(A_{r}-A_{i2}\right){\left(u_{02}-u_{r}\right)}^{2}\right]. \end{array}$$

Since the fluid of the receiving hole flows to the surface of the receiver, the volume flow rate in the left receiving hole is given by

(52) $$\begin{array}{c} q_{L}=C_{dr}A_{r}\sqrt{\frac{2}{\rho }\left(P_{2}-P_{r2}\right)}. \end{array}$$

Hence, the pressure acting on the left end of the spool is given by

(53) $$\begin{array}{c} P_{2}=P_{r2}+\frac{q_{L}^{2}\rho }{2C_{dr}A_{r}}. \end{array}$$

Based on the principle of flow continuity, the velocity of the reflected flow *u*_02_ is given by

(54) $$\begin{array}{c} u_{02}=\frac{u_{j}\cos\theta_{r}A_{i2}+u_{r}A_{r}}{A_{r}-A_{i2}}. \end{array}$$

Substituting Equation (51) into Equation (53), *P*_2_ is given by

(55) $$\begin{array}{c} P_{2}=\rho \left[\frac{A_{i2}{\left(u_{j}\cos\theta_{r}+u_{r}\right)}^{2}}{A_{r}-A_{i2}}+\frac{q_{L}^{2}}{2C_{dr}A_{r}}\right]. \end{array}$$

Due to the neglect of fluid compressibility, the load flow can be expressed as

(56) $$\begin{array}{c} q_{L}=A_{r}u_{r}. \end{array}$$

From Equations (47), (53), and (56), the load pressure applied on the two ends of the spool is expressed as

(57) $$\begin{array}{c} P_{L}=\frac{2\rho u_{j}^{2}}{A_{r}}\alpha_{a1}x_{j}-\frac{4\rho u_{j}u_{r}\cos\theta_{r}}{A_{r}}A_{1}\left(0\right)+\frac{2\rho u_{r}\cos\theta_{r}}{A_{r}}\alpha_{a1}x_{j}. \end{array}$$

When the JPS valve works, the nozzle is near the zero position. Then the pressure gain can be written as

(58) $$\begin{array}{c} k_{p}=\frac{\Delta P_{L}}{\Delta x_{j}}=\frac{8C_{dj}^{2}P_{s}}{A_{r}}\alpha_{a1}. \end{array}$$

Similarly, the flow gain can be written as

(59) $$\begin{array}{c} k_{q}={\left(1-\psi \lambda_{j}\right)}^{2}C_{d}C_{dj}A_{r}\sqrt{\frac{2P_{s}\cos\theta_{r}A_{j}}{\rho r_{j}A_{r}}}. \end{array}$$

Equation (57) can be rewritten as

(60) $$\begin{array}{c} P_{L}=k_{p}x_{j}-k_{q}q_{L}. \end{array}$$

#### 3.3.4. Liquid Flow Torque Acting on the Nozzle

When the fluid is injected into the receiver, part of the fluid will reflect and impact on the nozzle to form a liquid flow torque. As shown in Figure 7, as the nozzle has displacement *x*_*j*_, the reflected flow in the left and right receiver impact on the nozzle at velocity *u*_02_ and *u*_01_, respectively. According to the turbulent jet theory, the velocity of the reflected flow impacting on the nozzle can be written as

(61) $$\begin{array}{c} \left\{\begin{array}{c} u_{m1}=u_{01}\sqrt{\frac{H_{1}}{2b_{01}}}2.77\sqrt{1-\exp\left(-38.5\right)},\\ u_{m2}=u_{02}\sqrt{\frac{H_{2}}{2b_{02}}}2.77\sqrt{1-\exp\left(-38.5\right)}, \end{array}\right. \end{array}$$

where *u*_*m*1_ and *u*_*m*2_ are the velocity of the reflected flow impacting on the nozzle, respectively. *H*_1_ and *H*_2_ are the distance between the center of the left and right receiving holes and the nozzle, respectively. *b*_01_ and *b*_02_ are the width of annular reverse liquid flow of left and right receiving holes, respectively.

Within *dt* time, the mass of the reflected flow impacting on the nozzle is, respectively, given by

(62) $$\begin{array}{c} \left\{\begin{array}{c} dm_{m1}=\rho \left(A_{r}-A_{i1}\right)u_{m1}\text{d}t,\\ dm_{m2}=\rho \left(A_{r}-A_{i2}\right)u_{m2}\text{d}t. \end{array}\right. \end{array}$$

The reflected flow impinging on the nozzle from the left and right receiving holes forms reverse flow forces *F*_*m*1_ and *F*_*m*2_, respectively. The reverse flow forces are given by the momentum theorem.

(63) $$\begin{array}{c} \left\{\begin{array}{c} F_{m1}=\frac{dm_{m1}u_{m1}-dm_{01}u_{01}}{dt},\\ F_{m2}=\frac{dm_{m2}u_{m2}-dm_{02}u_{02}}{dt}. \end{array}\right. \end{array}$$

The angle between the force acting on the nozzle and the vertical direction is *θ*_*r*_. Then the horizontal resultant force *F*_*hon*_ and the vertical resultant force *F*_*per*_ of the force acting on the nozzle can be, respectively, written as

(64) $$\begin{array}{c} \left\{\begin{array}{c} F_{hon}=\left(F_{m1}-F_{m2}\right)\sin\theta_{r}\\ F_{per}=\left(F_{m1}-F_{m2}\right)\cos\theta_{r}. \end{array}\right. \end{array}$$

Substituting Equations (34), (35), (40), (46), (54), (61), (62), and (63) into Equation (64), the horizontal resultant force *F*_*hon*_ becomes

(65) $$\begin{array}{c} F_{hon}=\rho \left(u_{j}A_{i1}-u_{r}\cos\theta_{r}A_{r}\right)\left[\left(k_{h1}^{2}-1\right)\frac{u_{j}A_{i1}-u_{r}\cos\theta_{r}A_{r}}{A_{r}-A_{i1}}-u_{r}\cos\theta_{r}\right],\\ \;-\rho \left(u_{j}A_{i2}-u_{r}\cos\theta_{r}A_{r}\right)\left[\left(k_{h2}^{2}-1\right)\frac{u_{j}A_{i2}-u_{r}\cos\theta_{r}A_{r}}{A_{r}-A_{i2}}-u_{r}\cos\theta_{r}\right], \end{array}$$

where $k_{h1}=\sqrt{H_{1}/2b_{01}}2.77\sqrt{1-\exp\left(-38.5\right)}$ and $k_{h2}=\sqrt{H_{2}/2b_{02}}2.77\sqrt{1-\exp\left(-38.5\right)}$.

According to Equation (65), when *x*_*j*_ ∈ [−0.1,  0.1] mm, the relation curve between *F*_*hon*_ and *x*_*j*_ is shown in Figure 8. Figure 8 reveals that the relationship between *F*_*hon*_ and *x*_*j*_ is linear, and the formula is given by

(66) $$\begin{array}{c} F_{\text{flow}}=f_{hon}=k_{m}x_{j}, \end{array}$$

where *k*_*m*_=9.631 × 10^4^ N/m.

Since the distance between the vertical resultant force *F*_*per*_ and the gravity center of the armature is nearly zero, the torque generated by this force is neglected. Otherwise, the distance between the horizontal resultant force *F*_*hon*_ and the gravity center of the armature is *r*sin*θ*_*r*_. Then the flow torque generated by the force *F*_*hon*_ can be expressed as

(67) $$\begin{array}{c} T_{flow}=k_{m}x_{j}r\cos\theta_{r}. \end{array}$$

### 3.4. Spool Valve

When the fluid flows into the spool valve chamber and through the control window of the valve, the flow force acting on the spool is generated due to the change of fluid flow momentum caused by the change of flow velocity and direction. The flow force can be written as [11]

(68) $$\begin{array}{c} F_{y}=0.43Wx_{v}P_{s}, \end{array}$$

where *W* is the width of the spool valve window and *x*_*v*_ is the displacement of the spool.

Then the kinetic equation of the spool valve is given by

(69) $$\begin{array}{c} P_{L}A_{v}=m_{v}\frac{d^{2}x_{v}}{dt^{2}}+B_{v}\frac{dx_{v}}{dt}+f_{v}+F_{y}+F_{f}, \end{array}$$

where *A*_*v*_ is the effective area of the spool valve, *m*_*v*_ is the mass of the spool, *B*_*v*_ is the damping coefficient, and *f*_*v*_ is the friction.

Based on the principle of flow continuity, the flow in the spool valve can be written as

(70) $$\begin{array}{c} q_{L}=A_{v}\frac{dx_{v}}{dt}. \end{array}$$

## 4. Numerical Simulation

### 4.1. Spring Coefficient of the Feedback Rod

Due to the complex structure of the feedback rod, the spring coefficient *K*_*f*_ cannot be obtained by analytical solution. Then the FEA is utilized to calculate the spring coefficient. Since the force generates between the tube and the feedback rod, and the tube is fixed to the armature, the calculation of spring coefficient needs to consider the interaction between them. Based on the three dimensional model in Figure 3, the statics is adopted to analyze the spring coefficient by using ANSYS statics module. Firstly, the meshes are formed, as illustrated in Figure 9(a). The center of rotation is fixed, the counterclockwise rotation direction is specified as positive, and the force applied on the bottom of rod is specified as positive to the left. Then the material properties are defined as follows: the Young's modulus is 1.3e11 N/m^2^, the Poisson's ratio is 0.35, the density is 8230 kg/m^3^, and the yield strength is 1.128e9 *N*/*m*^2^. Finally, one of the displacement nephograms under different forces is shown in Figure 9(b).

From the numerical results, the relationship between the force applied on the rod and the rod's displacement is shown in Figure 10, and the relationship can be fitted by using the least square method.

(71) $$\begin{array}{c} F_{f}^{\prime }=0.00251x_{v}+0.04. \end{array}$$

From Equation (71), the stiffness of the rod can be written as

(72) $$\begin{array}{c} K_{f}=\frac{2.5e3N}{m}. \end{array}$$

### 4.2. Numerical Model of the Prestage

The fluid domain of the prestage refers to the jet tube, nozzle, receiver, and two ends of the spool, as shown in Figure 11. The high-pressure oil entering from the upper end of the jet tube is ejected from the nozzle, and then shoots into the two receivers to promote movement of the spool. The shape of the space between receiver and nozzle is disk, and the periphery of the space is connected with the oil return port of the JPS valve. Therefore, the fluid domain between the receiver and the nozzle is extracted into the shape of a disk, as illustrated in Figure 12.

As shown in Figure 12, the inlet and outlet are set as pressure inlet and pressure outlet boundary conditions, which are 21 MPa and 0.5 MPa, respectively. The number 15 hydraulic oil with the density of 839.3 kg/m^3^ and the kinetic viscosity of 13.84 mm^2^/s at 40°C is utilized as the working fluid. The grid independence is investigated to verify that the relative error of the computational meshes with 0.28 million cells is 0.1% compared to the finest grid with 1.2 million cells. Therefore, the computational meshes with 0.28 million cells are chosen for the rest computation.

Due to dynamic mesh technology of the software FLUENT, the FLUENT is adopted to calculate the transient flow field distribution of the prestage. The turbulence is predicted by the RNG *k* − *ε* model. As result, the value of *y* + should be less than 10.

The actions of the prestage affecting the flow field distribution mainly include the rotation of the nozzle and the movement of the spool. When the armature drives the nozzle to rotate clockwise an angle corresponding to the current input into the torque motor, the pressure difference deriving from the kinetic energy of the jet flow drives the spool to move. Since the end of the feedback rod is fixed in the center of the spool, the movement of the spool makes the nozzle embedded in the feedback rod rotate counterclockwise until the force acting on the spool is balanced. Then the movement of the prestage's flow domain consists of the rotation of the nozzle and the linear motion of the spool.

Because the force and torque exerted by the armature on the nozzle drive the nozzle to rotate, the effect of the force and torque on the nozzle is regarded as a rotation angle *θ*_*a*_. Taking the center of mass of the spring tube as the center of rotation, the displacement *x*_*g*_ can be considered as zero. Meanwhile, the nozzle is subjected to the force and torque exerted by the feedback rod. From Equations (9), (11), (13), and (14), the dynamic equation of nozzle is given by

(73) $$\begin{array}{c} T_{j}=J_{r}{\overset{¨}{\theta }}_{a}+B_{r}{\dot{\theta }}_{a}+\left[K_{21}r_{1}+K_{22}+K_{f}\left(r+b\right)\right]\theta_{a}+K_{f}x_{v}-k_{m}x_{j}r\cos\theta_{r}. \end{array}$$

The driving force of the spool can be obtained by integrating the fluid grid force on the both ends of the spool, which is given by

(74) $$\begin{array}{c} F_{p}=\int_{A_{1}}p_{i}dA-\int_{A_{2}}p_{j}dA=\sum_{M}p_{i}A_{i}-\sum_{N}p_{j}A_{j}, \end{array}$$

where *p*_*i*_ and *p*_*j*_ are the pressure applied on the mesh grid of the two ends of the spool, respectively, *A*_*i*_ and *A*_*j*_ are the areas of the mesh grid of the two ends of the spool, respectively, and *M* and *N* are the number of the mesh grid of the two ends of the spool, respectively.

From Equations (62) and (67), the dynamic equation of the spool is given by

(75) $$\begin{array}{c} \sum_{M}p_{i}A_{i}-\sum_{N}p_{j}A_{j}=m_{v}{\overset{¨}{x}}_{v}+B_{v}{\dot{x}}_{v}+f_{v}+F_{y}+F_{f}. \end{array}$$

Then, the dynamic relationship between the nozzle and the spool is described in Equations (46) and (48), and these equations can be used to define the motion of the nozzle and the spool by writing a user-defined function (UDF). Due to the rigid body characteristics of the nozzle and the spool, the DEFINE_CG_MOTION function can be utilized to describe the rotation of the nozzle and the translation of the spool. When the initial angle *θ*_*a*_ is set to 0.3° clockwise, the movement process of the nozzle and the spool can be obtained by the computational flowchart of the flow field in the prestage is shown in Figure 13. In each time step, the torque acting on the nozzle and the forces applied on the spool are calculated. Then the annular velocity and the translational velocity are computed to define the motion of the nozzle and the spool in the next time step, respectively.

## 5. Hierarchical Encourage Particle Swarm Genetic Algorithm

### 5.1. Structure of the Algorithm

GA has a strong global search ability, but its convergence speed is slow. Conversely, PSO draws on experience of previous iterations and converges more easily, but is prone to lose the diversity of population. To make full use of the advantages of GA and PSO in the same status, this study promotes a novel hybrid optimization method based on the hierarchical encourage idea which is from the concept of staff welfare system. Firstly, the employees are divided into three parts which consist of elite employees, excellent employees, and general employees based on the performance in the year-end assessment. Then the elite employees are encouraged by the higher salary to maintain their enthusiasm for work, followed by the excellent employees. By contrast, the general employees acquire the lowest salary. Meanwhile, the elite employees and the excellent employees are less likely to be eliminated. In addition, to maintain the competitiveness of employees, the salary is adjusted based on the next year-end performance.

Figure 14 shows the structure diagram of the proposed HEPGA algorithm. The majority of population are general individuals with GA, which improves the global search ability for the optimization algorithm. And the PSO algorithm provides the accurate local search for a few elite individuals and excellent individuals to maintain their superiority. Also, the different mutation rates are applied to protect the elite individuals and the excellent individuals, while eliminating the general individuals. The main body of algorithm is GA which guaranteeing the diversity of the population.

The steps of the proposed HEPGA algorithm are presented as follows:

Step 1: the parameters of the algorithm are initialized in this step. The parameters comprise the population size, elite rate (*r*_*el*_), excellent rate (*r*_*ec*_), crossover rate (100%), initial position (*x*_*ij*_), initial velocity (*v*_*ij*_), maximum velocity (*v*_max_), velocity control factors (*c*_1_=*c*_2_=2), inertia weight (*w*_*o*_), elite mutation rate (*δ*_*m*1_=0.005), excellent mutation rate (*δ*_*m*2_=0.008), general mutation (*δ*_*m*3_=0.01), and maximum number of iteration (*N*).
Step 2: the individuals of the population are initialized.
Step 3: the fitness values are calculated and utilized to guide the sorting of particles.
Step 4: according to the sorted population, the elite individuals *N*_*e*1_ and the excellent individuals *N*_*e*2_ are selected.
  (76) $$\begin{array}{c} N_{e1}=r_{el}\times N_{p},\\ N_{e2}=r_{ec}\times N_{p}-N_{e1}. \end{array}$$
Step 5: the updated equations of the particles' velocities and positions are given by
  (77) $$\begin{array}{c} x_{ij}\left(t+1\right)=x_{ij}+v_{ij}\left(t+1\right),\\ v_{ij}\left(t+1\right)=w\cdot v_{ij}\left(t\right)+c_{1}r_{1}\left[p_{ij}\left(t\right)-x_{ij}\left(t\right)\right]+c_{2}r_{2}\left[p_{gj}\left(t\right)-x_{ij}\left(t\right)\right]. \end{array}$$
where *p*_*ij*_ is the optimal location of individual, and *p*_*gj*_ is the global optimal location for all the individuals.
Step 6: the crossover operation is applied to the general individuals *N*_*e*3_ by using the following equations:
  (78) $$\begin{array}{c} N_{e3}=N_{p}-N_{e1}-N_{e2},\\ p_{1}^{1}=\frac{1}{2}\left[\left(1-\beta \right)p_{1}+\left(1+\beta \right)p_{2}\right],\\ p_{2}^{2}=\frac{1}{2}\left[\left(1+\beta \right)p_{1}+\left(1-\beta \right)p_{2}\right], \end{array}$$
where *p*_*i*_^*i*^ is generation *i*, *p*_*i*_ is the selected parent, and *β* is a random variable.
Step 7: the new generation from step 5 and step 6 is mutated by using different mutation rates.
Step 8: the parameters of population are updated.
Step 9: the algorithm will return to step 3 until the number of iteration equals the prespecified value.

### 5.2. Algorithm Evaluation

The effectiveness of the novel algorithm is investigated by using the Rosenbrock function, which is given by

(79) $$\begin{array}{c} f_{100}=\sum_{i=1}^{n-1}\left(100{\left(x_{i+1}-x_{i}^{2}\right)}^{2}+{\left(1-x_{i}\right)}^{2}n\right)=100. \end{array}$$

The search space of the Rosenbrock function is (−2.048,  2.048)^*n*^, and the global optimal value of this function is 0. Due to the unconstrained optimization characteristic and narrow bottom shape of the Rosenbrock function, the optimal value is difficult to be reached. Hence, the performance of the HEPGA is compared to PSO, GA-PSO, and HGP in reference [30]. The same PSO algorithm parameters are applied in the four optimization methods, and the mutation rate of the general group mentioned in Section 5.1 is used for GA-PSO and HGP. Meanwhile, HEPGA and HGP share the same elite rate. Also, the four optimization methods share the same population size that is 500, and the same maximal number of iterations is 1000.

To compare fairly and to eliminate the error caused by initializing the population, the four optimization methods share same initialization population and carry out 50 optimization calculations. After optimization, this paper utilizes the same criterion as in reference [30] to evaluate the HEPGA's effectiveness.  Table 1 and Figure 15 show the criterion comparison and convergence comparison, respectively. PSO and GA-PSO plunge into a local minimum, which is far from the optimal value. Although, the HGP algorithm reaches a global minimum value, which is almost 10 times greater than the global minimum value obtained by the HEPGA. This is because the HEPGA divides the population more finely and utilizes different mutation rates. Therefore, the proposed hybrid optimization algorithm can acquire the smaller global optimal value of the Rosenbrock function, which verifies the algorithm's effectiveness.

## 6. Experimental Platform

To verify the accuracy of the mathematical model of the JPS valve established by combining the numerical simulation and the theoretical formula, an experimental comparison is carried out. As shown in Figure 16, the experimental equipment includes pump system, oil pipeline, pressure sensor, pressure gauge, JPS valve, and signal acquisition devices. The pump system can supply constant pressure, and the supply oil pressure is set as 21 MPa. The pressure of supply oil, return oil, and pipelines is displayed in the pressure gauges. The pressure sensors are arranged at both ends of the spool to test the pressure data, and the data is compared to the results obtained by the mathematical model of the JPS valve. The model of the pressure is FYB26, the range of which is 0–35 MPa, the accuracy of which is ±2%. The step response of the optimized JPS valve is compared with that of the prototype.

## 7. Results and Discussion

### 7.1. Modification of the Mathematical Model

Although the submerged free jet stream is considered in the mathematical model, the influence of vortex on the dynamic characteristics of the JPS valve is neglected. From the computational flowchart in Figure 13, the diagrams of the velocity vector at four moments from movement to equilibrium of the spool are shown in Figure 17. The vortex exists in the space between the nozzle and the two receiving holes, which will prevent the jet flow from entering the receiving hole and decrease energy transfer efficiency. Also, the influence of the spool's movement on the flow field distribution affects its dynamic characteristics. As shown in Figure 18(a), the pressure in the left end of the spool is much larger than that in the right end at the beginning moment 0.03 ms. The large differential pressure drives the spool to move towards right direction quickly, and the rapid motion squeezes the fluid in the right end of the spool towards the receiving hole. Hence, the high-pressure region will exist in the receiving hole, as shown in Figure 18(b). Due to the rapid movement of the spool and the obstruction of the vortex to the jet flow, negative pressure will appear in the left end of the spool. Then the driving force applied on the spool is reversed, which causes the spool to decelerate. When the velocity of the spool decreases to a certain extent, the pressure in the left end of the spool will be greater than that in the right end, as illustrated in Figure 18(c). Hence, the driving force moves the spool to accelerate to the right direction until the force applied on the spool is equilibrium, as shown in Figure 18(d).

Therefore, the mathematical model of the prestage needs to be modified based on the numerical results. From Equations (60), (62), and (63), the transfer function between *θ*_*a*_ and *x*_*v*_ is given by

(80) $$\begin{array}{c} \frac{x_{v}\left(s\right)}{\theta_{a}\left(s\right)}=\frac{k_{p}A_{v}r}{m_{v}s^{2}+\left(B_{v}+k_{q}A_{v}^{2}\right)s+0.43WP_{s}}. \end{array}$$

Hence, the step response comparison of the spool's displacement is shown in Figure 19(a). Figure 19(a) shows that the step response of the mathematical model has overshoot, which do not appear in the numerical simulation. Then the mathematical model of the prestage is modified as follows:

(81) $$\begin{array}{c} \frac{x_{v}\left(s\right)}{\theta_{a}\left(s\right)}=\frac{0.8\cdot k_{p}A_{v}r}{m_{v}s^{2}+0.85\cdot \left(B_{v}+k_{q}A_{v}^{2}\right)s+0.43WP_{s}}. \end{array}$$

As shown in Figure 17(b), the step response is basically consistent with the results of the numerical simulation.

### 7.2. Optimization of the JPS Valve

In general, the adjustment time and overshoot of system's dynamic performance are required to be as small as possible. However, the adjustment time *t*_*s*_ and the overshoot *σ*_*se*_ of the jet pipe servo valve are in conflict. In other words, the reduction of the adjustment time increases the overshoot.

The structure parameters of the JPS valve affect its dynamic performance. From Equations (6), (16), and (62), these structure parameters apparently include the air gap *g*, distance *a*, theta *θ*_*r*_, diameter *D*_*j*_, diameter *D*_*r*_, and distance *l*_*j*_. To achieve convergence as soon as possible, the value range of these structure parameters is limited, as tabulated in Table 2.

The adjustment and the overshoot are two significant performance indexes that need to be considered simultaneously in system design, which can be regarded as two objective functions.

(82) $$\begin{array}{c} \left\{\begin{array}{c} \min F_{2}\left(\overset{⟶}{x}\right)=\left[\sigma_{se}\left(\overset{⟶}{x}\right)\right],\\ \min F_{3}\left(\overset{⟶}{x}\right)=\left[t_{ses}\left(\overset{⟶}{x}\right)\right]. \end{array}\right. \end{array}$$

The weight can be used to process the multiobjective function into a unified objective value, which can be written as

(83) $$\begin{array}{c} F_{se}\left(\overset{⟶}{x}\right)=\left[\frac{\sigma_{se}\left(\overset{⟶}{x}\right)}{\sigma_{se-\max}\left(\overset{⟶}{x}\right)},\;\frac{t_{se}\left(\overset{⟶}{x}\right)}{t_{se-\max}\left(\overset{⟶}{x}\right)}\right]\cdot {\overset{⟶}{w}}_{se}, \end{array}$$

where the $F_{se}\left(\overset{⟶}{x}\right)$ is the unified objective function, $\sigma_{se-\max}\left(\overset{⟶}{x}\right)$ is the maximum value of the overshoot, $t_{se-\max}\left(\overset{⟶}{x}\right)$ is maximum value of the adjustment time, and ${\overset{⟶}{w}}_{se}$ is the weight vector. The weight vector includes the weight of the overshoot *w*_*σ*_ which is set as 0.5, and the weight of the adjustment *w*_*t*_ which is set as 0.5. According to the technical index requirements, the values of $\sigma_{se-\max}\left(\overset{⟶}{x}\right)$ and $t_{se-\max}\left(\overset{⟶}{x}\right)$ are 0.11 and 0.015 s, respectively.

Since the optimization objectives are overshoot and adjustment time, the transfer function of the JPS valve needs to be obtained firstly. From Equations (15) and (66), the transfer function can be expressed as

(84) $$\begin{array}{c} \frac{x_{v}\left(s\right)}{i_{c}\left(s\right)}=\frac{K_{t}\left(m_{a}s^{2}+B_{a}s+K_{f}+K_{11}\right)}{K_{s6}s^{6}+K_{s5}s^{5}+K_{s4}s^{4}+K_{s3}s^{3}+K_{s2}s^{2}+K_{s1}s+K_{s0}}, \end{array}$$

where

(85) $$\begin{array}{c} K_{s5}=\frac{0.85J_{r}m_{a}m_{v}}{0.8k_{p}A_{v}r}\\ K_{s5}=\frac{0.85J_{r}m_{a}\left(B_{v}+k_{q}A_{v}^{2}\right)+m_{v}\left(J_{r}B_{a}+B_{r}m_{a}\right)}{0.8k_{p}A_{v}r}\\ K_{s4}=\frac{0.43J_{r}m_{a}WP_{s}+0.85\left(B_{v}+k_{q}A_{v}^{2}\right)\left(J_{r}B_{a}+B_{r}m_{a}\right)}{0.8k_{p}A_{v}r}\\ K_{s3}=\frac{0.43WP_{s}\left(J_{r}B_{a}+B_{r}m_{a}\right)+0.85\left(B_{v}+k_{q}A_{v}^{2}\right)\left(J_{r}K_{f}+J_{r}K_{11}+B_{r}B_{a}\right)+m_{v}\left\{B_{r}\left(K_{f}+K_{11}\right)+B_{a}\left[K_{21}r+K_{22}+K_{f}{\left(r+b\right)}^{2}-K_{\theta }\right]\right\}}{0.8k_{p}A_{v}r}\\ K_{s2}=\frac{0.43WP_{s}\left(J_{r}K_{f}+J_{r}K_{11}+B_{r}B_{a}\right)+0.85\left(B_{v}+k_{q}A_{v}^{2}\right)\left\{B_{r}\left(K_{f}+K_{11}\right)+B_{a}\left[K_{21}r+K_{22}+K_{f}{\left(r+b\right)}^{2}-K_{\theta }\right]\right\}+m_{v}\left[K_{21}r+K_{22}+K_{f}{\left(r+b\right)}^{2}-K_{\theta }\right]\left(K_{f}+K_{11}\right)}{0.8k_{p}A_{v}r}\\ \;+K_{f}\left(r+b\right)m_{a}\\ K_{s1}=\frac{0.43WP_{s}\left\{B_{r}\left(K_{f}+K_{11}\right)+B_{a}\left[K_{21}r+K_{22}+K_{f}{\left(r+b\right)}^{2}-K_{\theta }\right]\right\}}{0.8k_{p}A_{v}r}+K_{f}B_{a}\left(r+b\right)\\ K_{s0}=0.43WP_{s}\left(K_{f}+K_{11}\right)\left[K_{21}r+K_{22}+K_{f}{\left(r+b\right)}^{2}-K_{\theta }\right]+K_{f}\left(r+b\right)\left(K_{f}+K_{11}\right). \end{array}$$

The structure parameters in Table 2 are optimized based on the transfer function of the JPS valve and the HEPGA algorithm with the settings as tabulated in Table 3.  Figure 20 shows the flowchart of the JPS valve optimal design. After the initialization, the overshoot and the adjustment time are obtained by the step response of the input current 40 mA, and other procedures are same as the settings in Section 5.

As shown in Figure 21, the value of the objective function keeps decreasing with the increment of the iterations. As the number of iterations is 273, the objective function reaches the minimum value 0.937. The objective function reaches the local minimum 0.947 when the number of iterations is 169, and breaks the local minimum successfully. Because the value of the air gap *g* reaches the minimum 0.4 mm as the number of iterations is 273, the objective function increases with the number of iterations. As a result, the structure parameters are the optimal in the case where the number of iterations is 273. Then the optimal parameters are tabulated in Table 4, and the prototype is shown in Figure 22.

### 7.3. Experimental Verification

To verify the mathematical model of the JPS valve and compare the optimization results, the experimental device shown in Figure 16 is utilized to test the step response and frequency response of the optimal prototype. Since the experimental device can acquire the pressure of the control cavity at both ends of the spool valve, the step response of the spool's displacement *x*_*v*_ can be obtained by Equations (15), (57), (60), (66), (67), and (69).

Figure 23 shows the step response of the spool's displacement *x*_*v*_ under different inputs. The inlet pressure 21 MPa and outlet pressure 0.5 MPa under normal working condition are used as the input pressure of the mathematical model and experiment, and the input current is set as 10 mA, 20 mA, 30 mA, and 40 mA. Compared with the mathematical model before optimization, the dynamic characteristics of the optimized mathematical model have been significantly improved. As shown in Table 5, compared with that before optimization, the adjustment times of the JPS valve after optimization are, respectively, reduced by 26%, 27.8%, 29.3%, and 30.2% when the input current is 40 mA, 30 mA, 20 mA, and 10 mA. Under the same input current condition, the overshoot after optimization is reduced by 51.4%, 52.6%, 54.4%, and 57%, respectively.

In addition, the step response comparison of the optimized mathematical model and the experiment shows that the error of the adjustment time is 2.7%, 4.3%, 7.4%, and 7.1%, respectively, when the input current is 40 mA, 30 mA, 20 mA, and 10 mA. And the error of the overshoot is 1.3%, 6.1%, 5.7%, and 4%, respectively, under the same input current condition. This is because the compressibility of fluid is neglected and the overflow area of the two receiving holes is linearized in the mathematical model. Nevertheless, the step response of the simulation is considered to be similar to that of the experiment, which verifies the accuracy of the mathematical model and the effectiveness of the optimization algorithm based on HEPGA.

## 8. Conclusion

This paper proposes a more accurate mathematical and a novel hybrid optimization algorithm to improve the dynamic performance of the JPS valve. The main works of this paper are as follows:

1. Based on the turbulent submerged free jet theory, the mathematical model of the jet pipe servo valve is established. To improve the accuracy of the mathematical model, the CFD and the FEA approaches are adopted. In the CFD simulation, the dynamic mesh technique is utilized to analyze the flow field distribution in the actual working condition, and the numerical results are used to modify the mathematical. While for the FEA application, the stiffness of the feedback rod is obtained by static analysis.
2. Due to the conflict of overshoot and adjustment time in the dynamic performance, the HEPGA is proposed in this paper. Though the Rosenbrock verification, the HEPGA has better convergency than other PSO-GA hybrid methods. Then the HEPGA is used to optimize the main structure parameters of the JPS valve to minimize the overshoot and the adjustment.
3. Eventually, the experimental platform is utilized to test the step response of the prototype in the case where the input current is 10 mA, 20 mA, 30 mA, and 40 mA. The comparison results show that the adjustment time and the overshoot are reduced by 24.28% and 51.39%, respectively, compared with the JPS valve before optimization. Meanwhile, the comparison results show that the maximum error between the mathematical model and the experimental results is 6.09%, which verifies the mathematical model.

## Figures and Tables

**Figure 1:** Structure diagram of the JPS valve.

**Figure 2:** Magnetic flux diagram.

**Figure 3:** 3D diagram of the armature assembly.

**Figure 4:** Schematic diagram of the jet pipe amplifier.

**Figure 5:** Flow field structure of submerged free jet stream.

**Figure 6:** The comparison between the linear model and the nonlinear model of the flow area.

**Figure 7:** Schematic diagram of EMMP.

**Figure 8:** Diagram of relationship between the displacement of nozzle and the reverse force.

**Figure 9:** FEA of the feedback rod: (a) mesh and (b) displacement nephogram.

**Figure 10:** The relationship between force and displacement.

**Figure 11:** Three dimensional model of the prestage.

**Figure 12:** Flow domain and grid of the prestage: (a) computational domain and (b) grid.

**Figure 13:** Computational flowchart of the transient flow field.

**Figure 14:** Structure diagram of HEPGA algorithm.

**Figure 15:** Convergence comparison of four optimization algorithm.

**Figure 16:** Experimental platform: (a) schematic diagram; (b) jet pipe servo valve and sensor; (c) pump system; and (d) signal acquisition device.

**Figure 17:** The diagrams of the velocity vector at moment: (a) 0.03 ms; (b) 0.15 ms; (c) 1.0 ms; and (d) 27.03 ms.

**Figure 18:** The velocity distribution and pressure distribution of the prestage at moment: (a) 0.03 ms; (b) 0.15 ms; (c) 1.0 ms; and (d) 27.03 ms.

**Figure 19:** Comparison of spool displacement step response between mathematical model and numerical simulation: (a) comparison before modification and (b) comparison after modification.

**Figure 20:** Flowchart of the JPS valve optimal design.

**Figure 21:** Convergence of the JPS valve optimal design.

**Figure 22:** Prototype of the JPS valve.

**Figure 23:** Comparison of the step response: (a) 10 mA; (b) 20 mA; (c) 30 mA; and (d) 40 mA.

**Table 1:** Criteria comparison of optimization on Rosenbrock function.

Algorithm	Minimum evaluation	Average evaluation	Variance	Average time (min)
PSO	9.71e+1	9.91 *e*+1	1.45e+1	176
GA-PSO	9.73e+1	1.01e+2	5.59e-1	248
HGP	2.12e-7	3.73e-4	3.78e-3	265
HEPGA	2.1e-8	3.2e-5	3.11e-4	269

**Table 2:** The value range of the structure parameters.

Structure parameter	Value range
*g* (mm)	0.4∼0.5
*a* (mm)	10∼30
*θ*_*r*_ (°)	12∼20
*l*_*j*_ (mm)	0.1∼0.5
*D*_*r*_ (mm)	0.25∼0.5
*D*_*j*_ (mm)	1.0∼1.3

**Table 3:** Value of optimization parameter.

Optimization parameter	Value
Population size *N*_*p*_	100
Number of iterations *N*	300
Elite rate *R*_*ne*1_	0.2
Excellence rate *R*_*ne*2_	0.2
Mutation rate of elite individuals *δ*_*m*1_	0.005
Mutation rate of excellent individuals *δ*_*m*2_	0.008
Mutation rate of general individuals *δ*_*m*3_	0.01
Crossover rate	100%

**Table 4:** Structure parameters of the optimal design.

Structure parameter	Value
*g* (mm)	0.4
*a* (mm)	22.3
*θ*_*r*_ (°)	14
*l*_*j*_ (mm)	0.247
*D*_*r*_ (mm)	0.4
*D*_*j*_ (mm)	1.2

**Table 5:** Comparison of step response under different currents.

Input current (mA)	Overshoot %			Adjustment time (ms)		
	Before optimization	After optimization	Experiment	Before optimization	After optimization	Experiment
40	21	10.2	10.33	19.2	14.2	14.6
30	19.8	9.39	10	18.7	13.5	14.1
20	18.4	8.39	8.9	17.7	12.5	13.5
10	17.9	7.68	8	16.9	11.8	12.7

## Data Availability

All data and models generated or used during the study are included in the article.
